This article has been retracted.

# Berberine Inhibits Herpes Simplex Virus 1 Replication in HEK293T Cells

**DOI:** 10.1155/2022/7137401

**Published:** 2022-10-14

**Authors:** Yujuan Cui, Liangjun Zhang, Dandong Hu, Yingli Yang

**Affiliations:** ^1^School of Life Science, Northwest Normal University, Lanzhou, Gansu 730070, China; ^2^Beijing Yanqing Center for Diseases Prevention and Control, Beijing 102100, China; ^3^Beijing Yanqing Market Supervision Inspection and Testing Monitoring Center, Beijing 102100, China

## Abstract

Berberine exhibits polytrophic medicinal roles in various diseases and is safe and effective. However, its role and the underlying mechanism in the replication of herpes simplex virus 1 (HSV-1) remain unreported. This research aimed to determine the functional mechanisms of berberine on HSV-1 infection. We determined the CC50 (405.11 ± 15.67 *μ*M) and IC50 (45.6 ± 6.84 *μ*M) of berberine on HEK293T cells infected with HSV-1. Berberine inhibited the transcription and translation of HSV-1 activity-related genes (gD, ICP-4, ICP-5, and ICP-8) in HSV-1-infected HEK293T cells dose-dependently. Berberine also inhibited the phosphorylation of MAPK proteins (JNK and p38) and inflammatory responses induced by HSV-1 infection in HEK293T cells dose-dependently. In conclusion, berberine attenuates HSV-1 replication through its activity, infective ability, and inflammatory response. Our research indicated that berberine may be a candidate drug for HSV-1 infection.

## 1. Introduction

Herpes simplex virus (HSV) is a virus with double-stranded DNA under an envelope structure. HSV usually infects the body through the mucous membranes, skin, nerve tissue, and other related lesions. It has two serum subsets, HSV-1 and HSV-2. Infection with HSV-1 mainly leads to pharyngitis, cold sores, and keratitis and in severe cases will cause sporadic encephalitis and other dangerous diseases. HSV-2 mainly invades through damaged skin and mucous membranes to cause genital herpes [1]. Immediate early gene (*α* gene), early gene (*β* gene), and late gene (*γ* gene) express after HSV-1-infected host cells [2]. Infection cell protein (ICP4) expression peaks 2~4 hours after infection. The expression of the *β* gene requires activation of *α* gene products [3]. ICP5 and ICP8 can regulate viral DNA replication and participate in *γ* gene transcription [4]. Glycoprotein D (gD) is a late protein encoded by the *γ* gene peaking 12~15 hours after infection, which is the main component of the virus envelope and helps the virus to absorb and enter the host cell [5]. All these indicators can be used to evaluate the activity of HSV-1. Berberine is an alkaloid in the protoberberine group that existed in Berberidaceae, Papaveraceae, and Ranunculaceae [6].

Berberine shows polytrophic medicinal effects, including anti-inflammatory [7], antibacterial, and antifungal [8]. Berberine acts on a series of signaling pathways to improve diabetes [9–11]. Several *in vitro* studies have found that berberine diminishes the proliferation, migration, and metastasis of cancer cells and accelerates apoptosis [11–13]. It has been found that berberine promotes apoptosis by activating ROS-related signals, such as the JNK/p38 signaling pathway. ROS can activate JNK/p38 that block antiapoptotic protein Bcl-XL expression to release cytochrome C and stimulate caspases [14]. Recently, berberine shows antiviral properties against influenza A virus (IAV) [15], respiratory syncytial virus (RSV) [16], chikungunya virus (CHIKV) [17], enterovirus 71 (EV71, [18], human papillomavirus (HPV) [19], and herpes simplex 55 virus (HSV) [20], but its roles in HSV-1 infection is still unknown.

Here, we aimed to explore the antiviral and anti-inflammatory impact of berberine in HSV-1-infected HEK293T cells. It was reported that berberine can dose-dependently reduce the activity of HSV-1 and HSV-1-induced secretion of inflammatory factors and the phosphorylation of p38 and JNK.

## 2. Material and Methods

### 2.1. Material

#### 2.1.1. Cells

HEK293T cells were obtained from Fudan University (Shanghai, China) and kept in DMEM (Roche, Basel, Switzerland) plus 1% antibiotics and 10% FBS (Solarbio, Beijing, China) under a humid incubator containing 5% CO_2_ at 37°C.

#### 2.1.2. Drugs and Cell Treatments

Berberine was purchased from Solarbio (Beijing, China, purity ≥98%). HEK293T cells were grouped: control group, cells were untreated; HSV group, infected with 200 pfu/well HSV; HSV+5 *μ*M group, treated with 5 *μ*M berberine and 200 pfu/well HSV; HSV+10 *μ*M group, treated with 10 *μ*M berberine and 200 pfu/well HSV; HSV+15 *μ*M group, treated with 15 *μ*M berberine and 200 pfu/well HSV. Following 24-h culture, HEK293T cells were applied to plaque reduction assay, RT-qPCR, western blot, and ELISA.

## 3. Methods

### 3.1. Cytotoxicity Assay

The cytotoxicity of berberine on HEK293T cells was determined based on the CCK-8 assay [21]. The minimum berberine concentration required to produce a toxic effect on 50% of HEK293T cells (CC_50_) was calculated by regression analysis of the dose-response curve.

### 3.2. Plaque Reduction Assay

The anti-HSV-1 ability of berberine was evaluated [21] (Jung et al., 2011). In detail, HEK293T cells (1 × 10^5^/well) were cultured in a 24-well plate and treated with a corresponding dose of HSV-1 or berberine for 24 h. DMEM was added with 1% methylcellulose solution and 2% FCS (Solarbio, Beijing, China). Then, HEK293T cells were cultured under 5% CO_2_ at 37°C for 72 h. Monolayer cells were fixed and stained with 1% crystal violet, and formative plaques were counted. Finally, the minimum berberine concentration required to inhibit the 50% cytopathic effect (IC_50_) was calculated by regression analysis of the dose-response curve. The selectivity index (SI) was calculated by CC_50_/IC_50_.

### 3.3. RT-qPCR

RNA was isolated using TRIzol (Takara, Liaoning, China), and cDNA was obtained with M-MLV Reverse Transcriptase (RNase H) kit (Takara, Liaoning, China). RT-qPCR was performed according to the previous report [22].

### 3.4. ELISA

Following treatment with corresponding doses of HSV-1 or berberine for 24 h, 1 mL of extraction solution (Beyotime, Nanjing, China) was used to lyse HEK293T cells. Subsequently, the levels of inflammatory factors in the supernatant were determined with ELISA kits (Roche, Basel, Switzerland).

### 3.5. Western Blot

Proteins were obtained using Cell Lysis Buffer (Beyotime, Nanjing, China). Western blot was executed based on the previous description [23]. The primary antibodies were ordered from Roche (Basel, Switzerland 1 : 1000) and goat-anti-rabbit IgG secondary antibody was the secondary antibody (Santa Cruz, San Francisco, USA, 1 : 2000). OD was quantified by Image J (Image J Inc.).

### 3.6. Statistical Analysis

Data were presented as the mean ± SD of three independent experiments and processed by GraphPad 5.0 (GraphPad Software, Inc.). Student's *t*-test or one-way ANOVA plus Tukey post hoc tests were conducted. *P* < 0.05 indicated statistical significance.

## 4. Results

### 4.1. Berberine Antagonizes HSV-1 Infection in HEK293T Cells

Berberine's chemical structure formula was analyzed (Figure 1(a)), and CCK-8 assay was conducted to explore berberine cytotoxicity on HEK293T cells. The CC_50_ of berberine on HEK293T cells was calculated to be 405.11 ± 15.67 *μ*M, according to the regression analysis of the dose-response curve generated by CCK-8 assay (Figure 1(b)). In Figure 1(c), the IC_50_ of berberine on HEK293T cell infected with HSV-1 was 45.6 ± 6.84 *μ*M based on plaque reduction assay. The decrease in HSV-1 plaque formation caused by the increase in berberine concentration was dose-related, indicating that berberine could inhibit HSV-1 infection of HEK293T cells. The selective index (SI) was 7.43-10.86 (in Figure 1(d)).

### 4.2. Berberine Decreases HSV-1 Activity in HEK293T Cells

To further analyze the effects of berberine on HSV-1 activity in HEK293T cells, RT-qPCR and western blot analyses were followed to assess the levels of HSV-1 infection-related genes, including g D, ICP-4, ICP-5, and ICP-8. RT-qPCR manifested that HSV-1 upregulated the transcription of the four HSV-1 infection-related genes, relative to the control group (*P* < 0.01), while berberine antagonized this upregulation effect dose-dependently compared with the HSV group (Figure 2(a); *P* < 0.05). Consistently, HSV infection promoted g D, ICP-4, ICP-5, and ICP-8 protein expression, whereas berberine antagonized this promotion dose-dependently (Figure 2(b); *P* < 0.05). Taken together, berberine deceased HSV-1 activity in HEK293T cells.

### 4.3. Berberine Inhibits JNK and p38 Activation Induced by HSV-1 Infection

It has been revealed that HSV-1 activated the MAPK pathway [24, 25]. To further explore the effect of HSV-1 on the MAPK pathway, the phosphorylation levels of MAPK-related proteins (JNK and p38) in HEK293T cells were assessed. Results showed that HSV-1 infection upregulates the phosphorylation levels of JNK (*P* < 0.01) and p38 (*P* < 0.001) proteins. Besides, further investigation indicated that berberine inhibited the HSV-1 infection-induced phosphorylation levels of JNK and p38 in HEK293T cells dose-dependently (*P* < 0.05; Figure 3). Collectively, berberine inhibited JNK and p38 activation in HSV-1-treated HEK293T cells.

### 4.4. Berberine Decreases Inflammatory Responses Induced by HSV-1 Infection

HSV-1 triggers inflammatory responses, such as gingival stomatitis, cold sores, keratitis, and meningitis [26, 27]. To investigate the effect of berberine on inflammatory responses caused by HSV-1, RT-qPCR and ELISA were conducted. Our results showed that HSV-1 infection upregulated the mRNA and secretion levels of cytokines (*P* < 0.05) and berberine dose-dependently downregulated their levels triggered by HSV-1 infection (*P* < 0.05; Figures 4(a) and 4(b)). Taken together, berberine inhibited inflammatory responses induced by HSV-1 infection in HEK293T cells.

## 5. Discussion

Herpesviruses develop latency or cause oral and genital herpes, conjunctivitis, eczema herpeticum, and other diseases in 90% of the population. Herpesvirus also disturbs AIDS treatment under HIV infection [28]. It is important to seek drug candidates against HSV-1. Here, it was proved that berberine antagonized HSV-1 activity, inflammatory responses, and MAPK pathway activation in HEK293T cells which may contribute to the inhibition of HSV-1.

Berberine is cytotoxic to mast cells, rat hepatocytes, and Vero cells [17, 29, 30]. Cytotoxicity is a factor that must be considered in seeking a candidate for HSV-1 treatment. A study showed that berberine exerted an anticancer impact against HeLa cells with CC_50_ of 12.08 *μ*g/mL whereas exhibited low toxicity (CC_50_: 71.14 *μ*g/mL) on normal Vero cells [31]. Chin et al. found that the CC_50_ of berberine extracted from *Coptis chinensis* on Vero cells was 392.5 *μ*M, the IC_50_ was 66.49 *μ*M, and the SI was 5.9 [32]. Our results found that berberine could effectively inhibit HSV-1 activity (IC_50_: 45.6 ± 6.84 *μ*M) in HEK293T cells and was with low toxicity (CC_50_: 405.11 ± 15.67 *μ*M). The SI was 7.43-10.86, indicating berberine is a relatively safe and effective candidate for HSV-1 inhibition *in vitro*.

Our study found that HSV-1 infection upregulates the phosphorylation levels of JNK and p38 proteins, which was similar to other's reports. MAPK pathway activation was stimulated by HSV-1 infection [24, 25]. Berberine was illustrated to reduce the phosphorylation levels of JNK and p38 MAPK under CVB3 infection [33]. Zeng et al. illuminated the mechanism of berberine weakened host components JNK-MAPK, ERK-MAPK, and p38-MAPK activation [34]. Li et al. found that berberine retarded IL-33-stimulated cytokine production in RPMCs [29]. It has been demonstrated that the levels of ROS-related factors were boosted under IL-1*β* treatment and pretreatment of berberine exhibited inhibitory roles. Besides, the decrease in inflammatory responses indicated that berberine diminished the HSV-1 infection-caused inflammation.

In conclusion, our study showed that berberine inhibited HSV-1 replication by downregulation of HSV-1 activity, inflammatory responses, and MAPK pathway activation in HEK293T cells. Berberine may be a potential candidate for the treatment of HSV-1 infection.

## Figures and Tables

**Figure 1:** Berberine antagonizes HSV-1 infection in HEK293T cells. (a) Berberine chemical structure. (b) CCK-8 assay was performed to explore berberine CC_50_ in HEK293T cells. (c) Plaque reduction assay was carried out to explore berberine IC_50_ in HEK293T cells. (d) Plaque reduction assay was performed to assess the effect of berberine on HSV-1 plaque formation in HEK293T cells. All data are presented as the means ± SD.

**Figure 2:** Berberine decreases HSV-1 activity in HEK293T cells. (a) RT-qPCR was performed to assess the mRNA levels of HSV-1-related genes, including gD, ICP4, ICP5, and ICP8. (b) Western blot was performed to measure the protein levels of gD, ICP4, ICP5, and ICP8. All data are presented as the means ± SD. ^∗∗^*P* < 0.01*vs.* control group, ^#^*P* < 0.05*vs.* HSV group, ^∆^*P* < 0.05*vs.* HSV+5 *μ*M group, and ^+^*P* < 0.05*vs.* HSV+10 *μ*M group.

**Figure 3:** Berberine inhibits JNK and p38 activation induced by HSV-1 infection. Western blot was performed to assess the protein levels of p-JNK, JNK, p-p38, p38, and *β*-actin in HEK293T cells. All data are presented as the means ± SD. ^∗∗^*P* < 0.01 and^∗∗∗^*P* < 0.001*vs.* control group, ^#^*P* < 0.05*vs.* HSV group, ^∆^*P* < 0.05*vs.* HSV+5 *μ*M group, and ^+^*P* < 0.05*vs.* HSV+10 *μ*M group.

**Figure 4:** Berberine decreases inflammatory response induced by HSV-1 infection. (a) RT-qPCR analysis was performed to assess the mRNA levels of inflammatory cytokines, including IL-1*β*, IL-6, TNF-*α*, and IL-8 in HEK293T cells. (b) ELISA assay was carried out to assay IL-1*β*, IL-6, TNF-*α*, and IL-8 expression in HEK293T cell supernatant. All data are presented as the means ± SD. ^∗∗^*P* < 0.01 and^∗∗∗^*P* < 0.001*vs.* control group, ^#^*P* < 0.05*vs.* HSV group, ^∆^*P* <0.05 vs. HSV+5 *μ*M group, and ^+^*P* < 0.05 vs. HSV+10 *μ*M group.

## Data Availability

The data supporting the manuscript's conclusions will be made available to any qualified researcher without reservation.
